This article has been retracted.

# Side-by-Side Comparison of the Biological Characteristics of Human Umbilical Cord and Adipose Tissue-Derived Mesenchymal Stem Cells

**DOI:** 10.1155/2013/438243

**Published:** 2013-07-07

**Authors:** Li Hu, Jingqiong Hu, Jiajia Zhao, Jiarong Liu, Weixiang Ouyang, Chao Yang, Niya Gong, Luyang Du, Abhilasha Khanal, Lili Chen

**Affiliations:** ^1^Department of Stomatology, Wuhan Union Hospital, Tongji Medical College, Huazhong University of Science and Technology, No. 1277 Jiefang Avenue, Wuhan, Hubei 430022, China; ^2^Stem Cell Center, Wuhan Union Hospital, Tongji Medical College, Huazhong University of Science and Technology, Wuhan, Hubei 430022, China; ^3^Department of Gynaecology and Obstetrics, Wuhan Union Hospital, Tongji Medical College, Huazhong University of Science and Technology, Wuhan, Hubei 430022, China

## Abstract

Both human adipose tissue-derived mesenchymal stem cells (ASCs) and umbilical cord-derived mesenchymal stem cells (UC-MSCs) have been explored as attractive mesenchymal stem cells (MSCs) sources, but very few parallel comparative studies of these two cell types have been made. We designed a side-by-side comparative study by isolating MSCs from the adipose tissue and umbilical cords from mothers delivering full-term babies and thus compared the various biological aspects of ASCs and UC-MSCs derived from the same individual, in one study. Both types of cells expressed cell surface markers characteristic of MSCs. ASCs and UC-MSCs both could be efficiently induced into adipocytes, osteoblasts, and neuronal phenotypes. While there were no significant differences in their osteogenic differentiation, the adipogenesis of ASCs was more prominent and efficient than UC-MSCs. In the meanwhile, ASCs responded better to neuronal induction methods, exhibiting the higher differentiation rate in a relatively shorter time. In addition, UC-MSCs exhibited a more prominent secretion profile of cytokines than ASCs. These results indicate that although ASCs and UC-MSCs share considerable similarities in their immunological phenotype and pluripotentiality, certain biological differences do exist, which might have different implications for future cell-based therapy.

## 1. Introduction

Stem cells are self-renewable and capable of differentiating into at least two distinctive cell types. Mesenchymal stem cells (MSCs) are a population of stem cells, widely present in a large number of tissues including bone marrow, adipose tissue, umbilical cord blood and the cord itself, brain, liver, muscle, dental pulp, skin, and fetal tissues [1–6]. Owing to their multipotentiality, rapid proliferation, and strong capacities for self-renewal, mesenchymal stem cells hold great promise for tissue engineering and are therefore suitable seed cells for future cell therapy. Bone-marrow-derived MSCs (BMSCs) are the most commonly used MSCs for scientific and clinical purposes. Nevertheless, there are some limitations of BMSCs, such as the significant decrease in relative number of MSCs in the marrow and their differentiation potential with age [7]. In addition, the isolation procedure is invasive and may lead to complications and morbidity [8]; therefore it is necessary to find an alternative source of MSCs that have functions similar to the BMSCs but overcome these key limitations and portray a part of successful alternative.

In recent years, adipose tissue-derived mesenchymal stem cells (ASCs) and umbilical cord-derived mesenchymal stem cells (UC-MSCs) have been explored as new MSCs sources with obvious advantages over BMSCs [9, 10]. UC-MSCs are different from human umbilical cord-blood-derived mesenchymal stem cells (UCB-MSCs). Studies have shown that these MSCs, derived from Wharton's jelly tissue of the human umbilical cord, are actually better in many aspects than UCB-MSCs [11]. Both ASCs and UC-MSCs have drawn the attention of researchers due to their convenient harvesting procedures, excellent proliferation and differentiation abilities, less susceptibility to contamination of tumor cells, and no ethical restrictions. Various characteristics of ASCs and UC-MSCs have been studied, and many aspects focusing on their potential application in wound repair, tissue reconstruction, and disease treatment have been investigated [12–14]. But so far very few direct comparative studies focusing on these two types of cells have been made. We therefore designed a side-by-side comparative study. In consideration to keep uniformity of tissue sources and internal factors, we compared ASCs and UC-MSCs derived from the same donor. To this end, MSCs were isolated from the adipose tissue and umbilical cord from mothers delivering full-term babies, and thus side-by-side comparisons among various biological aspects including their in vitro cell culture dynamics, immunological phenotypes, multidifferentiation, proliferation and antiapoptic abilities, and their cytokine expression profiles were made.

We found that although ASCs and UC-MSCs share considerable similarities in their immunological phenotype and multipotentiality, certain biological differences do exist, including their adipogenesis, neurogenesis capability, and cytokine secretion profiles, which might have different implications for future cell-based therapy. 

 To our knowledge, very few side-by-side comparisons among various biological aspects were made between ASCs and UC-MSCs derived from the same individual. We believe that our finding will aid in future decision making in choosing the most suitable seed cell for cell-based therapy.

## 2. Material and Methods

### 2.1. Isolation and Culture of ASCs and UC-MSCs

 Human subcutaneous adipose tissues and umbilical cords were obtained from mothers (18–30 years old) planning on cesarean sections after obtaining written informed consent and approval by the Ethics Committee of Wuhan Union Hospital. ASCs and UC-MSCs were, respectively, isolated according to the procedures described by Bunnell et al. [15] and Seshareddy et al. [16]. Briefly, samples were washed with phosphate-buffered saline (PBS, Hyclone) to remove red blood cells. The adipose tissue was chopped into small pieces of about 25–50 mm^3^ and digested with 0.1% collagenase type I (Gibco) at 37°C for 60 min. The single cell suspension was obtained by filtering the digested material through a 100 *μ*m mesh filter to remove tissue debris. The ASC-containing cell suspension was centrifuged at 1000 rpm for 5 min, and the pellet was resuspended in specific MSC culture medium (Cyagen). 

The umbilical cord was transected longitudinally along the umbilical cord blood vessels. After careful removal of these blood vessels using forceps, Wharton's jelly tissue was chopped into small pieces of 1 mm^3^ and treated with 0.1% collagenase type I for 16 hours at 37°C and then washed and treated with 2.5% trypsin (Gibco) for 30 min at 37°C with agitation. Finally, ASCs and UC-MSCs were cultured in proliferation medium and seeded in 25 cm^2^ flasks (Costar) at a density of 5 × 10^7^ cells/mL. After 48–72 h incubation, nonadherent cells were removed by medium changing. Around 5–7 days after seeding, the cells reached 80% confluency. These cells were passaged using trypsinization. Cells at culture passage P3–P7 were used in the following studies. 

### 2.2. Flow Cytometry

Cultured ASCs and UC-MSCs at passage 3 were trypsinized (0.25% trypsin-EDTA), washed twice with PBS (PH = 7.4), and suspended in PBS at a concentration of 5 × 10^6^/mL, and then 1 mL sample was incubated with fluorescein isothiocyanate- (FITC-) conjugated monoclonal rabbit anti-human CD13, CD14, CD44, CD90, CD105, and CD34 (BD Biosciences) or isotype control for 30 min at 4°C according to the recommendation of the manufacturer. Finally, they were washed twice with PBS, centrifuged, and fixed in 4% paraformaldehyde. The stained cells were analyzed using a standard Becton-Dickinson FACSAria instrument and the CellQuest Pro software (BD Biosciences).

### 2.3. Growth Curves

In order to compare the growth curves of ASCs and UC-MSCs, the cells at passage 3 were trypsinized and modulated to the concentration of 2 × 10^4^/mL, and then the cells were seeded in 96-well plates (100 *μ*L/well, Costar). 24 hours later, 5 experimental wells and 1 control well were selected randomly to add CCK8 (10 *μ*L/well), and after 2-hour incubation, their absorbance values were tested by enzyme immunoassay analyzer, and the mean values were calculated. The growth curves were drawn after 9 successive days of continuous detection. 

### 2.4. Determination of Cells Antiapoptotic Ability

 In order to compare the antiapoptotic ability of ASCs and UC-MSCs, the cells at passage 3 were trypsinized and modulated to the concentration of 3 × 10^5^/mL, and then the cells were seeded in 6-well plates. Until 80% confluent, 1 × 10^−6^ mol/L dexamethasone was added, and the cells were collected by trypsinization after 48-hour incubation and then suspended in 500 *μ*L binding buffer, followed by adding 5 *μ*L Annexin V-FITC and 5 *μ*L Propidium Iodide. After incubation in the dark at room temperature for 5–15 min, the cells were analyzed by flow cytometry.

### 2.5. Multidifferentiation Ability Test of ASCs and UC-MSCs

 For adipogenic differentiation, ASCs and UC-MSCs were cultured in DMEM/F12 supplemented with 10% FBS, 1 mM dexamethasone, 0.5 mM methyl-isobutyl-xanthine, 10 mg/mL insulin, and 100 mM indomethacin (all from Sigma) for 3 weeks. At the end of the incubation, adipogenic differentiation was assayed by Oil-Red-O (Sigma) staining for lipid droplets.

 For osteogenic differentiation, ASCs and UC-MSCs were cultured in DMEM/F12 supplemented with 10% FBS, 0.1 mM dexamethasone, 10 mM b-glycerolphosphate, and 50 mM ascorbic acid (all from Sigma) for about 3 weeks. At the end of incubation, osteogenic differentiation was assayed by Alizarin red (Sigma) staining for calcium deposition. RNA was isolated from UC-MSCs and ASCs before and after the induction using Trizol reagent (Invitrogen, Carlsbad, CD, USA). cDNA was transcribed using Superscript III First Strand cDNA Synthesis kit following manufacturer's instructions (Invitrogen, Carlsbad, CD, USA). Quantitative real-time-PCR was performed with SYBR Green PCR reagents on an ABI Prism 7300 detection system (Applied Biosystems, Foster City, CA, USA). Beta-actin was used as an internal control. The normalized fold expression was obtained using the 2^−ΔΔCT^ method. Primers used for real-time PCR were summarized in Supplementary Table 1. (See Supplementary Material available online at http://dx.doi.org/10.1155/2013/438243).

For neurogenic differentiation, ASCs and UC-MSCs were cultured in either group A, DMEM/F12 supplemented with B27 (1 : 50) (Gibco), N2 (1 : 100) (Gibco), 20 ng/mL basic fibroblast growth factor (bFGF, Invitrogen), and 20 ng/mL epithelial growth factor (EGF, Invitrogen), or group B, DMEM/F12 supplemented with 5 *μ*mol/L retinoic acids (RA) for 6–10 days. The induction medium was refreshed every 3 days.

At the end of the induction period, neurogenic differentiation was assayed by immunofluorescence staining for neural and glial-specific protein expression. MSCs were washed with PBS and then incubated for 1 hour at room temperature with the following antibodies: rabbit anti-NSE mAb at final concentrations of 1/250 and mouse anti-GFAP mAb (Millipore, at final concentrations of 1/300), respectively. Primary antibodies were developed with secondary Dylight 488-goat anti-rabbit IgG and Dylight 546-rat anti-mouse IgG, both at final concentrations of 1/500. Secondary antibodies were incubated for 45 minutes at room temperature in the dark. After labeling, the cells were fixed with 0.4% paraformaldehyde and then covered with antifade mounting medium. Slides were immediately examined on a three-color immunofluorescence microscope (Nikon Instruments Inc.).

### 2.6. Preparation of ASC-CM and UC-MSC-CM and Protein Microarray Analysis of ASC-CM and UC-MSC-CM

 ASCs and UC-MSCs at passage 3 were cultured in specific mesenchymal stem cell growth medium until cells were approximately 80% confluent; the medium was replaced with serum-free DMEM/F12. Following incubation in serum-free medium for 48 h, the conditioned medium was collected, centrifuged at 1000 rpm for 5 minutes, and filtered through a 0.22 *μ*m syringe filter. ASC-CM and UC-MSC-CM were conserved at −20°C, and 5 mL medium was assayed by RayBio Biotin Label-based Human Antibody Array I (Cat no.: AAH-BLM-1-2, Norcross, GA, USA), which can detect the expression levels of 507 human proteins in cell culture supernatants simultaneously.

### 2.7. Statistical Analysis

 All values are expressed as mean ± SD. Comparisons between two groups were analyzed by Students' *t*-test and comparisons between more than two groups were analyzed by ANOVA. A value of *P* < 0.05 was considered statistically significant. All analyses were performed with SPSS 16.0.

## 3. Results

### 3.1. Morphologies of ASCs and UC-MSCs

Most of the primary ASCs adhered within 24 hours after plating and demonstrated polygonal or round morphology, and the cells stretched out pseudopodia and displayed similar fibroblast-like or spindle-shaped morphology around 2 days. ASCs proliferated rapidly within 5–7 days and gradually fused into a single layer, arranged in long spindle and distributed in clusters. The primary UC-MSCs began to adhere within 12 hours and formed scattered spindle morphology in 72 hours. UC-MSCs proliferated rapidly in 6–12 days and gradually fused into a sheet, parallel arrangement, and spiral-shaped distribution (Figure 1).

### 3.2. Flow Cytometry

 ASCs and UC-MSCs surface receptor molecules CD13, CD14, CD44, CD90, CD105, and CD34 were detected by flow cytometry. Results showed that ASCs and UC-MSCs both exhibited positive surface antigenicity for CD13, CD44, CD90, and CD105 and exhibited negative surface antigenicity for CD14 and CD34. Flow cytometry results are shown in Figure 2, and the expression of immunological phenotypes of ASCs and UC-MSCs is listed in Table 1. Statistical analysis showed that there was no significant difference in the surface antigenicity profiles of these two types of cells (*P* > 0.05).

### 3.3. Growth Curves

Growth curves of ASCs and UC-MSCs demonstrated that they had the following characteristics in common: in the first 12–18 hours, cells proliferated slowly and then entered the logarithmic growth phase, which continued for 5-6 days, and reached cell growth plateau in 7-8 days. The notable point was that their proliferation rates were basically the same in the first four days; however, UC-MSCs proliferated significantly faster than ASCs from the fifth day (*P* < 0.05). The results are shown in Figure 3.

### 3.4. Antiapoptotic Ability of ASCs and UC-MSCs

The flow cytometry results showed good antiapoptotic capacity of ASCs and UC-MSCs when induced by the high concentration of dexamethasone, which was not statistically different (*P* > 0.05).

### 3.5. Multidifferentiation Capabilities of ASCs and UC-MSCs

ASCs and UC-MSCs were able to efficiently differentiate into adipocytes and osteocytes. The adipogenesis of ASCs is much more prominent and efficient than that of UC-MSCs. ASCs changed to round-shaped adipocytes already around 2 days after induction, and at about 2 weeks, 95% of the ASCs were efficiently induced into adipocytes, whereas for UC-MSCs, clear morphology change began 5 days after induction and complete differentiation occurred three weeks after induction. The oil red staining for adipocytes is also more prominent for ASCs in comparison to UC-MSCs (Figure 4(a)). 

For osteogenic induction, UC-MSCs and ASCs from the same individual (passage 4) were cultured under osteogenic induction medium. Dramatic morphological changes already began 2 days after induction. At the end of two weeks, most MSCs already transformed from spindle-shaped MSCs to osteoblasts-like cells. Quantitative real-time PCR results were shown in Figure 5. As is shown, there was comparable significant upregulation of alkaline phosphatase, osteocalcin, and Runx2 in both UC-MSCs and ASCs. Osteocalcin is more significantly upregulated in UC-MSCs in comparison to ASCs, whereas alkaline phosphatase and Runx2 are more significantly upregulated in ASCs in comparison to UC-MSCs (Figure 5). Although no upregulation of leptin gene was identified, the equivalent upregulation of osteogenic genes of alkaline phosphatase, osteocalcin, and Runx2, together with equivalent Alizarin red staining (Figure 4(b)), suggests equivalence of osteogenic differentiation capacity for UC-MSCs and ASCs.

However, the differences were displayed (*P* < 0.05) in induction time and differentiation rate when they differentiated into neuron-like cells. We tried two induction methods: retinoid acid induction and neurobasal media induction. ASCs responded better to both methods. ASCs differentiated into neuron-like cells easily in culture medium of DMEM/F12 + B27 + N2 + bFGF + EGF (neurobasal media). Clear morphology changes begin as soon as two days after induction and became more prominent around 4-5 days. ASCs quickly lost their spindle-shaped morphology and displayed a bipolar or multipolar outlook. Neurites growth was most obvious around day 6, and multiple interconnections among cells can be seen. Longer cultivation in neurobasal medium (more than 10 days) leads to more prominent neurites outgrowth.

 Retinoid acid can induce ASCs into neurogenic differentiation as well. Clear morphology changes begin around 3 days after induction and became much more prominent around 5-6 days. Longer exposure (more than 10 days) and higher concentration (more than 5 uM) of retinoid acid lead to obvious cell death. The morphology of neurons induced by retinoid acid is significantly different from neurobasal media-induced neurons in that they are much smaller and usually display a spiky outlook (Figure 4). Interestingly, alone DMEM/F12 medium can induce ASCs to transform to neuron-like cells, similar to RA induction method (data not shown). The differentiation rate of ASCs is 38.6 ± 11.2% for neurobasal medium induction method and 45.5 ± 8.3% for RA induction method. The results are shown in Figure 4 and Table 2. 

Both conditions can induce UC-MSCs to differentiate into neuron-like cells as well but with a much lower efficiency (22.3 ± 4.8% for neurobasal medium induction method and 18.4 ± 5.6% for RA induction method (*P* < 0.01)). These results can be repeated in five individuals (Table 2).

### 3.6. Protein Microarray Analysis of ASC-CM and UC-MSC-CM

ASC-CM and UC-MSC-CM were assayed to determine the cytokines secreted by ASCs and UC-MSCs. Protein microarray analyses are shown in Figure 5; both these conditioned media contained a variety of cytokines. Signal value ratio of content in UC-MSC-CM and ASC-CM was used to analyze these cytokines, and statistical analysis had been carried out for those cytokines whose signal value exceeded 300, and the ratio was more than 1.5 or less than 0.66. The levels of expression of macrophage inflammatory protein 2 (MIP-2), interleukin 6 (IL-6), and growth-regulated oncogene (GRO) in UC-MSC-CM were significantly higher than those in ASC-CM, while the levels of expression of CD27 and neuregulin in ASC-CM were significantly higher than those of UC-MSC-CM. The results are shown in Figure 6 and Table 3.

## 4. Discussion 

Tissue engineering technology is one of the most promising means for solving difficult problems of tissues, organs defection, and wound healing [17, 18]. How to select suitable seed cells as well as their large-scale amplification has been an important issue for tissue engineering [19]. Adipose and umbilical cord tissues are good sources for mesenchymal stem cells, and both these cells have potential for multidifferentiation [20, 21]. In this study, we compared the similarities and differences between ASCs and UC-MSCs, aiming to provide a theoretical basis for clinical selection and application of seed cells. In consideration to keep uniformity of tissue sources and internal factors, we compared ASCs and UC-MSCs derived from the same donor.

In our study, we compared the cell morphologies and surface markers of mesenchymal stem cells from two different sources, the adipose and umbilical cord tissues. Two types of cells had similar morphologies and typical surface markers of MSCs, such as positive expression for CD13, CD44, CD90, and CD105 and negative expression for hematopoietic stem cells marker phenotypes of CD14, CD34, and there was no significant statistical difference in expression levels. The above results confirmed that, as mesenchymal stem cells, ASCs did not exhibit significant difference with UC-MSCs in the basic phenotypic characteristics of stem cells, which was consistent with the previous reports [22].

The proliferation and antiapoptotic abilities are very important for mesenchymal stem cells to maintain their characteristics of stem cells for long time in vitro. Related articles reported that ASCs and UC-MSCs both had strong self-renewal capacity [23, 24]. In this study, we in vitro cultured ASCs and UC-MSCs derived from the same individual and detected their proliferation ability. Their growth curves demonstrated that, compared with ASCs, UC-MSCs exhibited stronger proliferation ability, and the difference was significant (*P* < 0.05). The possible reason was that umbilical cord-derived cells might contain a lot of cytokines associated with the growth and development for neonatus, which could promote cell division and proliferation. Although UC-MSCs had stronger proliferation ability, in some of the existing reports, the proliferation ability of ASCs was superior to terminally differentiated cells and some other stem cells, and this ability basically met most of the experimental requirements [25]. Dexamethasone has biphasic effect on MSCs. In appropriate concentration (1 × 10^−9^ mol/L), dexamethasone can promote the osteogenic differentiation of MSCs [26], and there are also some studies which report that high concentration (higher than 1 × 10^−8^ mol/L) of dexamethasone could induce the apoptosis of MSCs [27]. So we chose 1 × 10^−6^ mol/L concentration of dexamethasone to induce apoptosis in this study, but our results showed that ASCs and UC-MSCs both had strong antiapoptotic ability, and there was no significant difference.

Multidifferentiation ability also is one of the factors for wide application of stem cells in tissue engineering field. There are many studies indicating that MSCs can differentiate into the three mesodermal cells in the appropriate induction environment [28]. The results of this study showed that both ASCs and UC-MSCs were able to efficiently differentiate into adipocytes and osteocytes. The adipogenesis of ASCs is much more prominent and efficient than that of UC-MSCs. We hypothesized that MSCs derived from different tissues still carry some of the reminiscent features of the original tissue. Some of the tissue-specific genes might already be and still are turned on, which might lead to the results we saw. 

We are particularly interested in neurogenic differentiation of both types of MSCs. We speculated that there must be some differences in the induction efficiency and in their response to different induction medium. We initially thought that UC-MSCs might respond better to neuronal induction since UC-MSCs had been widely used for treatment of neurological disorders with some noticeable clinical effects. But to our surprise, we found that ASCs responded much better to various induction methods than UC-MSCs. We tried two induction methods: retinoid acid (RA) induction and neurobasal medium induction. RA is a general differentiation and transdifferentiation agent for the generation of neurons [29]. It has been shown to induce the differentiation of cells during embryonic maturation into distinct organs, including the generation of neurons [30], whereas the culture medium of DMEM/F12 + B27 + N2 + bFGF + EGF is the medium generally used to produce neurospheres. These two induction methods had been reported in previous studies [31, 32]. We found that ASCs respond well to both methods. For neurobasal medium induction protocol, clear morphology changes begin as soon as two days after induction and became more prominent around 4-5 days. Neurites growth was most obvious around day 6, and multiple interconnections among cells can be seen. Retinoid acid can induce neuronal induction as well. Clear morphology changes begin around 3 days after induction and became much more prominent around 5-6 days. The neurons induced by retinoid acid are usually much smaller and usually display a spiky outlook. Interestingly, alone DMEM/F12 medium can induce ASCs to transform to a neuron-like cell, similar to RA induction method. Other papers have reported neural induction of UC-MSCs to various neuronal types. Here we failed to observe a prominent response of UC-MSCs to the above-mentioned induction methods. Our results suggested that, in the process of neuronal differentiation, ASCs might be more sensitive to different neuronal induction signals. These are probably due to the expression of multiple neurogenic genes that are already expressed in ASCs which might facilitate the neuronal induction process. However, further exploration of the exact mechanism for this phenomenon is necessary. 

The mechanisms of actions of stem cells on tissue regeneration and wound healing include two hypotheses [33, 34]: differentiation theory and paracrine theory, and the latter is more recognized, which means that stem cells can secrete a variety of cytokines acting on surrounding cells or migrate to tissue defect sites through cell homing, to participate in the reconstruction of tissues. ASC-CM and UC-MSC-CM contained a variety of cytokines secreted by cells [27]; we found that the types of cytokines were nearly the same in ASC-CM and UC-MSC-CM through protein microarray analysis, but the differences existed in expression levels of cytokines. The content of some cytokines varied greatly; for example, the expressions of MIP-2, IL-6, and GRO in UC-MSC-CM were significantly higher than those in ASC-CM, while the expressions of CD27 and neuregulin in ASC-CM were significantly higher than those in UC-MSC-CM. MIP-2 is the main chemotactic cytokine of neutrophil, and it can specifically promote neutrophil migrating to the inflammatory tissue, to get rid of pathogens and participate in the body's defense reaction [35]; MMP-1 is involved in mediation of a wide range of physiological and pathological processes in the body, such as the formation of embryo, tissue remodeling, wound healing, inflammation, and apoptosis [36]. IL-6 can promote the proliferation of a variety of cells, and this might be one of the reasons for UC-MSCs proliferating faster than ASCs [37]. In addition, IL-6 and IL-3 can synergistically promote cell differentiation, and in our protein microarray analysis results, the levels of expression of IL-3 in ASCs and UC-MSCs supernatants were similar (results not shown); therefore, in most aspects of differentiation, the capacity of two types of stem cells did not exhibit significant difference. As a member of NGFR/TNFR gene superfamily, CD27 is expressed in most of peripheral T cells and can be used as a second messenger with its ligand CD70 to promote T cells proliferation [38]. It is also involved in the process of T cells differentiation and the immune reaction of cells [39]. Neuregulin, a neuromodulation protein, is a kind of nutritional factor containing epidermal growth factor-like domain that plays an important role in nervous system development process [40]. Different contents of these cytokines indicated that suitable stem cells could be selected depending on the different needs in the tissue engineering fields.

## 5. Conclusion

In summary, the basic biological characteristics of mesenchymal stem cells derived from adipose and umbilical cord tissues are similar to each other, and both of them have strong self-renewal capacity, antiapoptotic capacity, and multidifferentiation capacity. The types of cytokines were nearly the same in ASC-CM and UC-MSC-CM, but there were differences in the levels of expression of certain cytokines. Interestingly, we found that ASCs responded much better to various neuronal induction methods in comparison to UC-MSCs. In consideration of the wide use of human umbilical cord-derived MSCs in stem cell therapy for treatment of neurological disorders, we suggest that human adipose mesenchymal stem cells may also be a valuable source for stem cell therapy in the future. 

## Supplementary Material

The Primer sequences (5'-3') used for Real-time PCR are listed in Supplementary Table 1.
Flow cytometric images of immunophenotyping with SSEA-PE antibody are shown in Supplementary Figure 1.

## Figures and Tables

**Figure 1:** Morphologies of ASCs and UC-MSCs cultured ex vivo. ((a)–(d)) Morphology of ASCs. (a) P0; (b) P1; (c) P2; (d) P3. ((e)–(h)) Morphology of UC-MSCs. (e) P0; (f) P1; (g) P2; (h) P3. Scale bar = 200 *μ*m. ASCs: adipose mesenchymal stem cell; UC-MSC: human umbilical cord mesenchymal stem cell, P: passage.

**Figure 2:** Immunophenotyping of ASCs and UC-MSCs. (a1)–(a4) Flow cytometry analysis of ASC; (b1)–(b4) flow cytometry analysis of UC-MSCs.

**Figure 3:** Proliferation and antiapoptotic ability of ASCs and UC-MSCs. (a) Growth curves of ASCs and UC-MSCs showed that UC-MSCs proliferated significantly faster than ASCs from the fifth day (*P* < 0.05). (b) Flow cytometric analysis of antiapoptotic ability of ASCs and UC-MSCs. (c) Statistical analysis of antiapoptotic ability of ASCs and UC-MSCs. Results showed that these two types of cells had good antiapoptotic capacity, and there was no significant difference (*P* > 0.05).

**Figure 4:** Multilineage differentiation of ASCs ((a1), (b1), (c1), and (d1)) and UC-MSCs ((a2), (b2), (c2), and (d2)). (a1) and (a2) Adipogenesis; (b1) and (b2) osteogenesis; (c1) and (c2) neurogenesis; (d1) and (d2) immunofluorescence staining of NSE for neurogenic differentiation. Scale bar = 100 *μ*m.

**Figure 5:** Relative quantification of osteogenic gene expression using real-time PCR after osteogenic induction in ASC and UC-MSCs. The mRNA levels were normalized using the expression of the reference gene (beta-actin). Results were from three independent experiments. ASC: adipose tissue-derived mesenchymal stem cells; UC-MSC: umbilical cord-derived mesenchymal stem cells.

**Figure 6:** Protein microarray analysis of ASC-CM (a) and UC-MSC (b) and changes of difference proportion of a variety of cytokines. Results showed that there were a lot of cytokines in ASC-CM and UC-MSC, and the contents of these cytokines were not exactly the same in two conditioned mediums, and the cytokines whose content had very obvious difference were MIP-2, IL-6, CRO, and MMP-1.

**Table 1:** Comparison of expression of surface markers of ASCs and UC-MSCs.

Antibody	ASCs (%)	UC-MSCs (%)	*P*
CD13	97.46 ± 1.97	96.81 ± 1.66	0.681
CD44	97.67 ± 1.55	97.51 ± 1.14	0.897
CD90	96.56 ± 1.21	98.03 ± 1.22	0.212
CD105	96.45 ± 0.91	97.18 ± 1.33	0.481
CD14	1.12 ± 0.13	0.96 ± 0.14	0.209
CD34	1.32 ± 0.30	1.10 ± 0.17	0.315

**Table 2:** Comparison of neurogenic differentiation of ASCs and UC-MSCs (*n* = 5).

Cell	DMEM/F12 + RA		DMEM/F12 + N2 + B27 + EGF + bFGF	
	Time (days)	Successful differentiation rate (%)	Time (days)	Successful differentiation rate (%)
ASCs	4.8 ± 1.3	45.5 ± 8.3	3.8 ± 2.2	38.6 ± 11.2
UC-MSCs	7.1 ± 2.1	18.4 ± 5.6	9.5 ± 2.2	22.3 ± 4.8
*P*	0.001	0.001	0.001	0.001

Results of neurogenic differentiation of ASCs and UC-MSCs are presented. ASCs responded better to both methods, exhibiting the higher differentiation rate and relatively shorter induction time than UC-MSCs in the same induction method.

**Table 3:** Proportion of some cytokines content in ASC-CM and UC-MSC-CM.

Cytokines	ASC-CM	UC-MSC-CM	UC-MSC-CM/ASC-CM
MIP-2	121.00	1,578.59	**13.05**
IL-6	194.50	1,329.72	**6.84**
GRO	303.00	1,433.86	**4.73**
MMP-1	501.00	1,599.55	3.19
IL-8	160.50	486.48	3.03
Thrombospondin-1	355.50	734.03	2.06
TIMP-2	408.00	778.37	1.91
Pentraxin3/TSG-14	352.00	661.00	1.88
Osteoprotegerin/TNFRSF11B	423.00	792.94	1.87
EG-VEGF/PK1	324.50	583.56	1.80
TRAILR4/TNFRSF10D	332.50	589.96	1.77
ENA-78	175.00	308.44	1.76
Vasorin	355.00	620.63	1.75
ErbB2	199.00	340.87	1.71
Decorin	333.00	570.32	1.71
Angiopoietin-2	267.50	447.65	1.67
IFN-beta	320.00	534.58	1.67
Flt-3 Ligand	245.00	403.09	1.65
FLRG	383.50	576.94	1.50
CXCR6	450.50	296.74	0.66
Activin RIA/ALK-2	393.00	253.94	0.65
D6	385.00	247.32	0.64
NRG3	1,328.50	804.41	0.61
Siglec-9	476.50	281.08	0.59
MMP-20	1,085.00	636.95	0.59
sFRP-3	622.00	359.18	0.58
CCR3	343.00	179.81	0.52
HCR/CRAM-A/B	1,261.00	604.52	**0.48**
Heregulin/NDF/GGF/Neuregulin	478.00	223.72	**0.47**
CD27/TNFRSF7	369.50	161.72	**0.44**

Part of cytokines were listed in table. Signal value of these cytokines was more than 300, and their content proportion in UC-MSC-CM and ASC-CM was more than 1.5 or less than 0.66. Results showed that the content of MIP-2, IL-6, and GRO in UC-MSC-CM was significantly more than that in ASC-CM, while the content of HCR, Heregulin, and CD27 in ASC-CM was significantly more than that in UC-MSC-CM.
